# Effect of the Kanghuier Transparent Hydrocolloid Dressing in Preventing Central Venous Catheter Infection and Phlebitis after Cardiac Surgery

**DOI:** 10.1155/2022/4700257

**Published:** 2022-04-01

**Authors:** Xiaoling Han, Jiayi Li, Ping Zeng, Chunfeng Luo, Dongmei Zhou

**Affiliations:** ^1^Department of Nursing, Zhuhai People's Hospital (Zhuhai Hospital Affiliated with Jinan University), Zhuhai, Guangzhou 519000, China; ^2^Department of Spine and Osteopathy, Zhuhai People's Hospital (Zhuhai Hospital Affiliated with Jinan University), Zhuhai, Guangzhou 519000, China; ^3^Department of Cardiothoracic Surgery, Zhuhai People's Hospital (Zhuhai Hospital Affiliated with Jinan University), Zhuhai, Guangzhou 519000, China; ^4^Department of General Surgery, Zhuhai People's Hospital (Zhuhai Hospital Affiliated with Jinan University), Zhuhai, Guangzhou 519000, China

## Abstract

**Background:**

As cardiac surgery is complicated, time-consuming, and traumatic, it may cause great damage to the patient's body. Therefore, postoperative indwelling venous catheters are required for hemodynamic monitoring and rapid fluid replenishment. Intravenous catheterization infection can easily lead to phlebitis, which not only affects the success of the operation and patient recovery but may also lead to death in severe cases. Good perioperative care is key to reducing postoperative infection in patients, and the choice of dressings for patients with catheterization plays an important role in reducing catheter infection.

**Objective:**

The Kanghuier transparent hydrocolloid dressing is known to effectively prevent and treat wound infections. This study is aimed at exploring whether it can reduce the incidence of postoperative catheter infection and phlebitis in patients undergoing cardiac surgery.

**Methods:**

A total of 196 patients undergoing cardiac surgery in the Department of Cardiothoracic Surgery of Zhuhai People's Hospital (Zhuhai Hospital Affiliated with Jinan University) from January 2020 to June 2020 were selected. Among them, 98 patients receiving Kanghuier transparent dressing intervention were selected as group A, and the remaining 98 patients receiving traditional sterile gauze intervention were selected as group B. The incidence of infection and related complications, phlebitis, inflammatory factors, pain at the infusion site, nursing comfort and satisfaction, and quality of life were analyzed and compared between the two groups.

**Results:**

It was found that compared with group B, the postoperative central venous catheter infection rate and the incidence of phlebitis were significantly lower in group A. In addition, the inflammatory response of patients in group A was better relieved. Moreover, the nursing comfort and satisfaction and the quality of life of patients in group A were significantly improved.

**Conclusion:**

This study suggests that the Kanghuier transparent hydrocolloid dressing is effective in the prevention and treatment of central venous catheter infection and phlebitis in patients after heart surgery.

## 1. Introduction

Cardiac surgery is characterized by complex operation, long duration, and great trauma, and a series of invasive operations, such as tracheal intubation anesthesia, arteriovenous catheterization, indwelling catheterization, and postoperative mechanical ventilation, are required during the operation, which cause serious damage to the body of patients [1, 2]. Although cardiopulmonary bypass is performed during surgery, surgical wounds can still severely weaken the patient's autoimmunity, predisposing heart surgery patients to a high risk of hospital infections [3]. In addition, most patients undergoing cardiac surgery have obvious cardiac insufficiency before surgery, which further increases the risk of postoperative infection [4]. The central venous catheter is directly connected to the cardiac vessels to monitor the central venous pressure of patients during the perioperative period and serve as an important channel for the delivery of vasoactive drugs [5, 6]. Therefore, indwelling central venous catheters are common and important in cardiac surgery. However, the postoperative nursing requirements for patients with indwelling central venous catheters are high. Leakage of fluid or blood at the catheter site due to improper care not only reduces the accuracy of central venous pressure measurement but also easily leads to bacterial invasion and infection [7, 8]. Postoperative central venous catheter infection not only affects the treatment effect but also increases the hospital stay and treatment costs of patients. Insufficiently controlled infections may lead to phlebitis, local redness, swelling, heat, and pain, as well as systemic symptoms such as fever and chills. In severe cases, phlebitis may develop into deep vein thrombosis or sepsis, which could easily lead to death [9, 10]. Therefore, the perioperative care of patients with indwelling central venous catheters after cardiac surgery is very important.

At present, the conventional prevention and treatment methods for postcardiac surgery patients against central venous catheter infection or phlebitis mainly include local sealing therapy, physical therapy, or local wet compress therapy [11]. However, it has been found in clinical practice that although these methods can reduce the incidence of infection and promote patient recovery to a certain extent, the procedures are difficult with high requirements for nursing staff and slow effects. Moreover, these methods limit the patients' range of motion and reduce their nursing comfort [12].

In recent years, a growing number of studies have shown that modern wound dressings are highly effective in the prevention and treatment of catheter-related infections [13–19]. A wide variety of dressings are currently available for use in catheter-related infections and phlebitis. Among them, the Kanghuier transparent dressing is a hydrocolloid dressing that can effectively prevent phlebitis with the characteristics of simple operation, good efficacy, and economic benefits, which has been proved to have a preventive effect on pressure ulcers and diabetic foot ulcers [20, 21]. However, more studies are needed to confirm whether it can play a role in the prevention and treatment of central venous catheter infection and phlebitis after cardiac surgery. In this study, we explore the role of hydrocolloid dressings in the prevention of central venous catheter infection and phlebitis in patients with indwelling central venous catheters after cardiac surgery, aiming to provide a reference for improving perioperative care and reducing postoperative infections in heart surgery patients.

## 2. Materials and Methods

### 2.1. Research Subjects

This retrospective study enrolled patients who underwent cardiac surgery in the Department of Cardiothoracic Surgery of Zhuhai People's Hospital (Zhuhai Hospital Affiliated with Jinan University) from January 2020 to June 2020. This research has been approved by the Ethics Committee of Zhuhai People's Hospital (Zhuhai Hospital Affiliated with Jinan University). Inclusion criteria were as follows: (1) patients aged 18-70 years; (2) patients who voluntarily participate in the study and cooperate throughout the process, with the informed consent provided; (3) patients with indwelling central venous catheters after heart surgery; (4) patients with follow-up treatment in our hospital after the operation; and (5) patients with no preoperative infection. Exclusion criteria were as follows: (1) unconscious patients and (2) patients with dysfunction of the liver, lung, kidney, and other vital organs. A total of 196 patients meeting the above criteria were included, and according to the treatment methods, they were divided into group A (Kanghuier transparent dressing; *n* = 98) and group B (traditional sterile gauze; *n* = 98). After comparison, it was found that there were no significant differences in general demographic data and medical history between the two groups, suggesting that both groups of patients are comparable for the purpose of observing our chosen variables, such as infection and related complications, phlebitis, and inflammatory factor levels (the general data distribution of patients is shown in Figures 1(a)–1(c)).

### 2.2. Care Methods

The postoperative care for both groups of patients was carried out by trained and licensed nursing staff. After the operation, 0.5% povidone-iodine was used for routine disinfection. Then, for patients in group A, the Kanghuier transparent dressing (Coloplast, Denmark, 10 cm × 10 cm, as shown in Figure 2(a)) was used to cover the puncture site and the skin proximal to the puncture vessel, with both the length and the width of the dressing 1 cm greater than the damaged skin. When applying the transparent covering, nurses ensured that there were no bubbles between the transparent patch and the skin and that the edges were flat. The dressing was changed once every 2–3 days, but if it became damp or the puncture site became infected, it was replaced immediately. Group B was covered with sterile gauze (Hubei Jinshida Medical Products Co., Ltd., 10 cm × 10 cm, as shown in Figure 2(b)) after routine disinfection. The covering method and precautions were the same as those for group A. Furthermore, cases of loosened gauze were replaced immediately.

### 2.3. Outcome Measures

#### 2.3.1. Determination of Central Venous Catheter Infection

Patients who met any two of the following three criteria were judged to have infections [22]. (1) The patient's body temperature increased significantly during catheterization and returned to normal or was greatly decreased after catheter removal. (2) The skin temperature at the catheterization site was significantly higher than that in other areas and was accompanied by redness, swelling, pain, and increased secretions, with positive bacterial culture results. (3) The patient's body temperature and white blood cell count increased significantly, and the bacterial culture results of blood or catheter specimens were positive. In addition, complications such as an ectopic catheter, catheter blockage, and skin allergy and blood oozing at the catheterization site were observed and recorded.

#### 2.3.2. Determination of Phlebitis

The study subjects were evaluated for phlebitis according to the guidelines for the occurrence and grading of phlebitis formulated by the Infusion Nurses Society [23], with the specific criteria shown in Table 1. Grade 0 indicated no occurrence of phlebitis, and grades 1 to 4 indicated the presence of phlebitis.

#### 2.3.3. Pain Assessment at the Infusion Site

After 1 day of catheterization, the patient's comfort level was assessed by the Visual Analogue Scale (VAS) [24, 25], with 0 being no discomfort, 1-3 being mild pain, 4-6 being moderate pain, 7-9 being severe pain, and 10 being extreme pain.

#### 2.3.4. Comparison of Inflammatory Factors

Approximately 5 mL of fasting venous blood was drawn from patients 3 days before, as well as 3 days, 7 days, and 10 days after cardiac surgery, respectively, to detect serum levels of interleukin-1*β* (IL-1*β*), interleukin-6 (IL-6), tumor necrosis factor-*α* (TNF-*α*), and interleukin-10 (IL-10) using the enzyme-linked immunosorbent assay (ELISA). The experiment procedure strictly followed the instructions of ELISA kits (Wuhan Fine Biotech Co., Ltd., EH3655, EH0201, EH0302, and EH0173). The specific procedures are as follows: the specific capture antibody globulin diluted with a coating buffer was treated with 3 hours of water bath at 37°C to remove the coated solution, followed by three rinses with a washing buffer. Then, the test sample containing the antigen was added to the plates, incubated, and washed. Then, the enzyme-labeled specific antibody was added, followed by the addition of the substrate to develop color. After incubation, the plates were washed, and the results were observed. Finally, the wavelength at 450 nm was detected by a microplate reader (Beijing ZEPING Bioscience & Technology Co., Ltd., 25-315S), and the concentration was calculated.

#### 2.3.5. Patient Care Comfort and Satisfaction

On the 10th day after surgery, the self-made nursing comfort questionnaire and nursing satisfaction questionnaire were used to evaluate patient comfort and satisfaction with nursing, respectively. Both questionnaires were conducted on a 10-point scale, with >9 indicating very comfortable/satisfied, 8-9 indicating relatively comfortable/satisfied, 6-7 indicating basically comfortable/satisfied, and <6 indicating uncomfortable/dissatisfied.

#### 2.3.6. Quality of Life Assessment

At discharge, the 36-Item Short-Form Health Survey (SF-36) [26] was used to evaluate the quality of life of patients from the dimensions of cognitive function, body function, role function, social function, and emotional function, with a score of 100. The higher the score, the better the quality of life.

### 2.4. Statistical Analysis

Data analysis and image rendering were performed using SPSS 25.0 (SPSS Inc., Chicago, IL) and GraphPad Prism 8.2 (GraphPad Software, USA), respectively. Quantitative data conforming to a normal distribution are represented as mean ± standard deviation; multigroup comparisons used one-way analysis of variance (ANOVA), and an SNA-Q test was used for pairwise comparisons. Qualitative data, expressed as frequencies and percentages, were analyzed using the chi-squared test. When the theoretical frequency was between 1 and 4, the chi-square was corrected. If the theoretical frequency was less than 1, the exact probability method was used to calculate the chi-square; the data were ranked and summed. Differences between datasets are considered significant when *P* < 0.05.

## 3. Results and Discussion

### 3.1. Central Venous Catheter Infection and Related Complications in Patients

The comparison of the incidence of catheter infection between the two groups showed that the incidence in group A which used the Kanghuier transparent dressing was only 16.33%, which was lower than that of 25.51% in group B (*P* < 0.05). A further comparison of the total complications showed that the total incidence of complications in group A was also significantly lower than that in group B (*P* < 0.05), as shown in Table 2 and Figure 3. These results indicate that the Kanghuier transparent dressing can reduce the risk of catheter infection and complications in patients with indwelling central venous catheters after cardiac surgery.

### 3.2. Occurrence of Phlebitis in Patients

By comparing the occurrence of phlebitis between the two groups, it can be found that the number of patients without phlebitis in group A was higher than that in group B. In addition, among the patients with phlebitis, most were grade 1 phlebitis in group A while grade 2 phlebitis in group B. Statistical analysis showed a significant difference in the occurrence of phlebitis between the two groups (*P* < 0.05), as shown in Table 3 and Figure 4.

### 3.3. Expression of Inflammatory Factors

No difference was found in the expression of inflammatory factors between the two groups three days before surgery. On the third day after surgery, the serum levels of IL-1*β*, IL-6, and TNF-*α* in both groups were higher than those before the operation, while the level of IL-10 was lower. This may be because the operation has caused greater trauma to the body, putting the body in a state of stress. However, the changes of IL-1*β*, IL-6, TNF-*α*, and IL-10 levels in group A were less significant than those in group B (*P* < 0.05). On the 7th and 10th days after the operation, the levels of IL-1*β*, IL-6, and TNF-*α* decreased in both groups, and the decrease in group A was greater than that in group B. The level of IL-10 increased, and the degree of increase in group A was higher than that in group B (*P* < 0.05), as shown in Table 4 and Figure 5.

### 3.4. Pain Assessment at the Infusion Site

By evaluating the pain degree at the infusion site, it was found that neither group had extreme pain, and most of the patients in the two groups were in mild pain. However, the total incidence of pain at the infusion site in group A was significantly lower than that in group B, and the difference was statistically significant (*P* < 0.05), as shown in Table 5 and Figure 6.

### 3.5. Patient Care Comfort and Satisfaction

The proportion of patients in group A who were very comfortable and very satisfied with the care were 42.86% and 48.98%, respectively, which were higher than those in group B (31.63% and 33.67%). There were significant differences in overall comfort and satisfaction between the two groups (*P* < 0.05), as shown in Table 6 and Figure 7.

### 3.6. Comparison of Patients' Quality of Life

The SF-36 scale was used to evaluate the quality of life of patients. It was found that the scores of cognitive, body, role, social, and emotional function in group A were higher than those in group B (*P* < 0.05), as shown in Figure 8.

## 4. Discussion

Central venous catheterization is a new technique commonly used in major surgical operations, which can monitor hemodynamics and replenish fluid quickly during and after the operation, with the characteristics of convenient operation and high safety [27]. However, cardiac surgery is very traumatic, and the patient's immune system is weakened after surgery. Central venous catheterization is an invasive operation that destroys the patient's skin barrier. If microorganisms invade the patient's body at the catheter site, infection and even phlebitis can occur [28–32]. Therefore, the nursing of the catheterization site is key to reducing the risk of postoperative catheter infection.

Hydrocolloid dressings are mainly composed of hydrophilic particles and hydrophobic polymers, which become hydrogels after absorbing wound exudate, and can promote the synthesis of cellular collagen and accelerate wound healing while protecting the skin against external bacterial invasion [33–35]. At the same time, the hydrocolloid dressing can promote skin metabolism at the patient's catheterization site, accelerate the proliferation of microvessels, and reduce the risk of phlebitis [36]. Zhai et al. found that a biocompatible composite hydrogel can improve the ability of cells to adsorb proteins, increase the self-repair ability of cells, and promote bone tissue regeneration [37]. Depan and Misra also reported that superhydrophilic and antibacterial dressings can reduce the incidence of wound infections [38]. Cai et al. also confirmed that a supramolecular hydrogel can reduce the damage from external stimuli to the skin of patients, thereby reducing the body's oxidative stress response [39].

In this study, we found that the incidence of venous catheter infection in patients using the Kanghuier transparent dressing was only 16.33%, which was significantly lower than that in patients using traditional sterile gauze (25.51%). Further comparison between the two groups showed that the total incidence of complications in patients who used the Kanghuier transparent dressing was also significantly lower than that in patients using traditional sterile gauze. This suggests that the Kanghuier transparent dressing can reduce the risk of catheter infection and complications in patients with indwelling central venous catheters after cardiac surgery. Comparing the occurrence of phlebitis between the two groups, we found that the incidence of phlebitis in group A was higher than that in group B; and in patients with phlebitis, most patients in group A had grade 1 phlebitis while grade 2 phlebitis in group B. These results show that the Kanghuier transparent dressing can reduce the risk of phlebitis in patients with indwelling central venous catheters after cardiac surgery.

Then, we compared the preoperative levels of inflammatory factors between the groups and found no significant difference between the two groups before the operation. However, we found that patients who used the Kanghuier transparent dressing had lower levels of inflammatory factors after the operation, while the anti-inflammatory factor (IL-10) level was raised. These results suggest that the Kanghuier transparent dressing can reduce postoperative inflammatory responses, which may also be the main reason for the low incidence of postoperative infection and phlebitis in patients from group A. In addition, we observed that the total incidence of pain at the infusion site in group A was significantly less than that in group B, which may be related to the better fixation and fewer dressing changes of the Kanghuier transparent dressing compared with traditional gauze.

As is known to all, cardiac surgery is characterized by complex operation, long duration, and great trauma, which will undoubtedly cause adverse emotions in patients, compromising their treatment compliance and even affecting the smooth treatment in serious cases [40, 41]. Therefore, appropriate care for patients is critical. The study found that group A was superior to group B in terms of comfort, nursing satisfaction, and quality of life. The reason behind this, we believe, is related to the following points: (1) the Kanghuier transparent tape reduces the incidence of catheter infection and phlebitis in patients; (2) the Kanghuier transparent dressing can effectively prevent severe pain in patients; and (3) the Kanghuier transparent dressing has good fixation and will not cause discomfort such as sultry heat and dampness. The novelty of this study is to confirm that the Kanghuier transparent dressing has a good clinical effect in central venous catheter infection and phlebitis after cardiac surgery from the aspects of infection and related complications, phlebitis, inflammatory factors, pain at the infusion site, nursing comfort and satisfaction, and quality of life, which provides a new and more excellent choice for the management of this patient population.

In view of the great damage caused by cardiac surgery to the body of patients, we also put forward the following nursing suggestions in addition to the application of the Kanghuier transparent dressing, hoping to provide a reference for the perioperative care of patients undergoing cardiac surgery [42–44]. (1) When choosing a central venous catheter, the catheter with high histocompatibility and smoothness should be selected to avoid the blood vessel wall damage and infection caused by the contact between the catheter and the patient's myocardial tissue. (2) Attention should be paid to the reasonable selection of a puncture site. At present, it is generally believed that the infection rate of the subclavian puncture is lower than that of the internal jugular venous puncture. Therefore, when using indwelling central venous catheters for cardiac surgery patients, the subclavian puncture should be given priority. (3) During catheterization, it is necessary to ensure that operators are skilled and strictly follow the principles of aseptic operation. At the same time, the puncture time should be shortened as much as possible to reduce damage to the patient's body. And after a successful puncture, the stability of catheter fixation should be ensured to avoid abnormal position or blockage due to loosening of the catheter. (4) Postoperative catheter indwelling time should be shortened as much as possible according to the actual situation of the patient. During intubation, close attention should be paid to the patient's puncture site, and the dressing should be changed regularly to ensure that the puncture site is dry and sterile. (5) If a patient develops an infection, a drug susceptibility test should be carried out in time to take targeted antibacterial treatment.

## 5. Conclusion

To sum up, the immune system of patients declines rapidly after cardiac surgery, resulting in a high risk of catheter infection and phlebitis. This study found that the incidence of central venous catheter infection and phlebitis in patients who used the Kanghuier transparent dressing after cardiac surgery was significantly reduced, and the body's inflammatory response was also greatly reduced. Furthermore, the Kanghuier transparent dressing can improve patients' nursing comfort, satisfaction, and quality of life to a certain extent. Therefore, we believe that while reducing the risk of venous catheter infection and phlebitis, the Kanghuier transparent dressing can improve nursing comfort and satisfaction in patients undergoing cardiac surgery.

## Figures and Tables

**Figure 1:** General information distribution of the two groups of patients. (a) The gender of patients in the two groups. (b) The age of patients in the two groups. (c) The surgical causes of patients in the two groups.

**Figure 2:** Dressings used in the postoperative care of patients. (a) Kanghuier transparent dressings used in group A. (b) Sterile gauze used in group B.

**Figure 3:** Comparison of infection and related complications.

**Figure 4:** Comparison of the incidence of phlebitis.

**Figure 5:** Expression of inflammatory factors in patients during the perioperative period. (a) Expression of IL-1*β*. (b) Expression of IL-6. (c) Expression of TNF-*α*. (d) Expression of IL-10. Comparison between the two groups, ^∗^*P* < 0.05.

**Figure 6:** Comparison of pain at the infusion site between the two groups.

**Figure 7:** Comparison of patient care comfort and satisfaction. (a) Nursing comfort. (b) Nursing satisfaction.

**Figure 8:** Scores of various dimensions of quality of life. (a) Cognitive function score. (b) Body function score. (c) Role function score. (d) Social function score. (e) Emotional function score. ^∗^*P* < 0.05.

**Table 1:** Phlebitis grading judgment standards.

Grade	Main symptoms
0	No obvious symptoms
1	Redness at the catheter site with slight pain
2	Redness at the catheterization site with obvious pain
3	Obvious redness and swelling at the catheterization site, cord-like veins can be palpated, accompanied by obvious pain
4	Pus exudates on the basis of grade 3, and the length of the cord-like vein exceeds 250 mm

**Table 2:** Comparison of infection and related complications.

Group	Infection	Ectopia	Obstruction	Irritability	Bleeding	Total complications
A (*n* = 98)	16 (16.33)	1 (1.02)	1 (1.02)	0	1 (1.02)	19 (19.39)
B (*n* = 98)	25 (25.51)	3 (3.06)	2 (2.04)	1 (1.02)	3 (3.06)	34 (34.69)
*χ* ^2^						5.069
*P*						0.024

**Table 3:** Comparison of the occurrence of phlebitis.

Group	0	1	2	3	4
A (*n* = 98)	87 (88.78)	9 (9.18)	2 (2.04)	0	0
B (*n* = 98)	77 (78.57)	8 (8.16)	12 (12.24)	1 (1.02)	0
*Z*	−2.122				
*P*	0.034				

**Table 4:** Comparison of inflammatory factor levels during the perioperative period.

Inflammatory factor	Grouping	Preoperation	Postoperation			*F*_time_
		3rd day	3rd day	7th day	10th day	
IL-1*β* (pg/mL)	A (*n* = 98)	12.74 ± 1.75	19.07 ± 2.14	15.22 ± 2.07	10.76 ± 1.58	597.004^∗^
	B (*n* = 98)	12.28 ± 1.66	20.18 ± 2.37	18.06 ± 1.97	14.92 ± 1.82	
	*t*	1.888	3.441	9.839	17.092	
	*P*	0.061	<0.001	<0.001	<0.001	

IL-6 (pg/mL)	A (*n* = 98)	14.62 ± 3.19	33.21 ± 8.06	21.68 ± 5.41	12.37 ± 2.97	502.411^∗^
	B (*n* = 98)	15.43 ± 3.64	35.49 ± 7.18	29.08 ± 6.74	21.49 ± 4.58	
	*t*	1.657	2.091	8.476	16.541	
	*P*	0.099	0.038	<0.001	<0.001	

TNF-*α* (pg/mL)	A (*n* = 98)	57.63 ± 8.05	97.18 ± 16.44	73.19 ± 15.71	59.81 ± 11.97	347.121^∗^
	B (*n* = 98)	56.22 ± 7.96	104.74 ± 19.62	89.57 ± 16.09	77.61 ± 13.08	
	*t*	1.233	2.924	7.211	9.938	
	*P*	0.219	0.004	<0.001	<0.001	

IL-10 (ng/mL)	A (*n* = 98)	11.69 ± 1.04	3.18 ± 0.57	7.09 ± 1.37	10.82 ± 1.96	1749.014^∗^
	B (*n* = 98)	11.43 ± 1.08	2.39 ± 0.51	6.19 ± 1.29	8.13 ± 1.65	
	*t*	1.717	3.236	4.735	10.391	
	*P*	0.088	0.001	<0.001	<0.001	

*Note.* ^∗^ *P* < 0.001.

**Table 5:** Comparison of pain at the infusion site between the two groups.

Group	Mild pain	Moderate pain	Severe pain	Extreme pain	Total incidence
A (*n* = 98)	16 (16.33)	3 (3.06)	0 (0.00)	0 (0.00)	19.39%
B (*n* = 98)	30 (30.61)	6 (6.12)	2 (2.04)	0 (0.00)	38.78%
*χ* ^2^					8.930
*P*					0.003

**Table 6:** Patient care comfort and satisfaction.

	Grouping	Score			
		>9	8–9	6–7	<6
Degree of comfort	A (*n* = 98)	42 (42.86)	36 (36.73)	19 (19.39)	1 (1.02)
	B (*n* = 98)	31 (31.63)	34 (34.69)	29 (29.59)	4 (4.08)
	*Z*	−2.182			
	*P*	0.029			

Degree of satisfaction	A (*n* = 98)	48 (48.98)	35 (35.71)	14 (14.29)	1 (1.02)
	B (*n* = 98)	33 (33.67)	41 (41.84)	23 (23.47)	1 (1.02)
	*Z*	−2.283			
	*P*	0.022			

## Data Availability

The simulation experiment data used to support the findings of this study are available from the corresponding author upon request.
